The article "Clinical Observation and Pharmacoeconomic Evaluations of Original Research Drug and Generic Drug Bortezomib in the Treatment of Multiple Myeloma" was retracted in 2023. Reasons: signs of a paper mill; suspected computer-generated content; unreliable results or conclusions; lack of ethics approval or compliance.

# Clinical Observation and Pharmacoeconomic Evaluations of Original Research Drug and Generic Drug Bortezomib in the Treatment of Multiple Myeloma

**DOI:** 10.1155/2022/5201354

**Published:** 2022-03-29

**Authors:** Yongchao Liang, Ying Zhu, Ying Zhang, Ziwei Chen, Boyang Li, Aijun Liu, Lihong Liu

**Affiliations:** ^1^Capital Medical University, Beijing 100069, China; ^2^Department of Pharmacy, Beijing Chao-yang Hospital, Capital Medical University, Beijing 100020, China; ^3^Jianguomen Community Health Service Center, Dongcheng District, Beijing 100005, China; ^4^Xiaotangshan Hospital, Beijing 102211, China; ^5^Department of Hematology, Beijing Chao-yang Hospital, Capital Medical University, Beijing 100020, China

## Abstract

**Background:**

Multiple myeloma (MM) is one of the hitherto incurable malignant blood tumors. Bortezomib plays an important role in the treatment of MM.

**Objective:**

We aimed to compare effectiveness, safety, and pharmacoeconomic evaluations of the original research drug and the generic drug Bortezomib in the treatment of MM, so as to provide a reasonable basis for the selection of drugs in clinical diagnosis and treatment.

**Methods:**

A collection of 374 patients with MM were diagnosed and treated with combined Bortezomib in our hospital from July 2019 to January 2020.Two hundred and sixty nine cases met the criteria for inclusion and discharge. According to the different drug manufacturers, divided into the original research drug group (*n* = 149) and the generic drug group (*n* = 120). The effectiveness and safety were separately counted, and use the cost-minimization analysis to make the pharmacoeconomic evaluations.

**Results:**

Compared with the results of the two groups, there was no statistical difference between the two groups of treatment efficacy or adverse reaction rates (*P* > 0.05). The average daily cost of the original research drug group was 2954.38 Chinese yuan (CNY), the average treatment cost per cycle was 32967.69 CNY, the average daily cost of the generic drug group was 2697.29 CNY, and the average treatment cost per cycle was 29129.57 CNY. The price of the generic drug group is lower than the original drug group, and there was a statistical difference between the two groups (*P* < 0.05).

**Conclusion:**

There was no difference between the two groups of effectiveness or safety, and the generic drug is more economical in the treatment.

## 1. Introduction

Multiple myeloma (MM) is caused by multiple locus plasma cells which proliferate abnormally in the bone marrow, resulting in multiple tissue and organ damage and making it one of the hitherto incurable malignant blood tumors [1, 2]. Bortezomib plays an important role in the treatment of MM. The importance of Bortezomib in various regimens of MM therapy is reflected in the guidelines of the International Myeloma Working Group, the US National Comprehensive *Cancer* Network, and the cellular and molecular genetics (mSMART) criteria established by the Mayo Clinic research group. However, the price of imported original research drug is very expensive, leading to a huge economic burden on patients. In this study, the efficacy and safety between original research drug and generic drug Bortezomib was compared based on an observational study. The pharmacoeconomic analysis was carried out to provide reasonable reference for variable alternative selection in clinical diagnosis and treatment, so as to make a little contribution for the early realization of “Value-based Healthcare” in China [3].

### 1.1. Aim of the Study

We aimed to compare effectiveness, safety, and pharmacoeconomic evaluations of the original research drug and the generic drug Bortezomib in the treatment of MM, so as to provide a reasonable basis for the selection of drugs in clinical diagnosis and treatment.

### 1.2. Ethics Approval

The study/data collection was conducted after approval by the Ethics Committee of Beijing Chao-yang Hospital, Capital Medical University (Approval reference number: 2019-4-15–4).

## 2. Methods

### 2.1. Inclusion and Exclusion Criteria

Patients with multiple myeloma treated with Bortezomib chemotherapy regimen in our hospital from July 2019 to January 2020 were followed up and collected. Inclusion criteria: (1) diagnosed MM, (2) with the result of FISH, and (3) treatment with Bortezomib. Exclusion criteria: (1) combined treatment with Bortezomib was less than 2 weeks, (2) insufficient clinical data, and it was unable to perform treatment efficacy and adverse reaction rates, and (3) both original research drug and generic drug were applied.

### 2.2. Study Subjects

There were 374 patients diagnosed with MM which was collected in this study. One case was of smoldering myeloma, 4 cases died within 2 cycles in the treatment, 7 cases with no Bortezomib in the treatment regimen, and 5 cases used both drugs. Eighty eight cases, whose treatment information was unable to be collected, were transferred to other hospitals or returned to local hospitals due to residential area and economic problems. According to inclusion and exclusion criteria, patients who met the criteria were 269 cases. They were divided into the original research drug group (*n* = 149) and the generic drug group (*n* = 120) based on the different drug manufacturers. Baseline date of patients were collected: gender, age, disease staging (ISS stage, traditional DS stage, and revised R-ISS stage) [4–6], and basic diseases (hypertension, diabetes, coronary heart disease, atrial fibrillation, cerebral hemorrhage, cerebral infarction, atherosclerosis, vein thrombosis of lower limb, hyperlipidemia, high uric acid hematic disease, hypothyroidism, thyroid nodules, chronic respiratory system disease, digestive system diseases, rheumatoid immune-related diseases, history of orthopaedical surgery, allergies, etc.). Test and examination information of patients before each cycle of treatment (blood routine, urine routine, biochemistry, blood *β*2 microglobulin, serum free light chain (FLC) test, serum immunofixation electrophoresis, serum M protein electrophoresis, 24-hour urine M protein, bone marrow puncture, bone marrow flow MRD test, etc.). All medical expenses incurred during hospitalization were collected.

### 2.3. Treatment Method

After diagnosing with MM, patients were treated with the chemotherapy regimen combined with Bortezomib. The recommended dose of Bortezomib was 1.3 mg/m^2^, subcutaneously injected twice weekly for two weeks (i.e., injected on days 1, 4, 8, and 11), followed by 10 days of withdrawal as a treatment cycle. The actual dose was appropriately reduced to 1.0 mg/m^2^ according to the tolerance level of patients or changed to once a week according to the tolerance level of patients, with continuous 4 weeks of administration (i.e., injection on the 1st, 8th, 15th, and 22nd days), followed by 13 days of withdrawal, namely, a treatment cycle. Continuous treatment for at least 2 cycles, followed up for 6 cycles. During the treatment, according to the condition and the occurrence of adverse reactions, timely symptomatic treatment, program adjustment, and drug dose adjustment were performed.

Drugs used: Bortezomib in the original research drug development group was VELCADE (manufacturer: BSP Pharmaceuticals S.p.A, specification: 3.5 mg/dose, approval no.: J20171067, and price: 5639.50 CNY/dose), and Bortezomib in the generic drug group was Xintai (manufacturer: Jiangsu Hausen Pharmaceutical Group Co., LTD., specification: 3.5 mg/branch, approval no.: National Drug Approval WORD H20173306, and price: 3929.20 CNY/branch).

Drugs for combined use include Lenalidomide (Remifamide) (Celgene Intenational Sarl, specification: 25 mg/tablet, approval no.: H20171348, and price: 1030.68 CNY/tablet), Lenalidomide (Zipuyi) (manufacturer: Qilu Pharmaceutical Co., LTD., specification: 25 mg/tablet, approval no.: National Drug Approval H20193115, and price: 182.8571 CNY/tablet), Thalidomide (manufacturer: Changzhou Pharmaceutical Co., LTD., specification: 25 mg/tablet, approval no.: National drug Approval H3202619, and price: 1.91 CNY/tablet), Cyclophosphamide (manufacturer: specification: 0.2 g/tablet, approval no.: H20160467, and price: 24.8 CNY/tablet), Dexamethasone (manufacturer: Tianjin Lisheng Pharmaceutical Co.,Ltd., specification: 0.75 mg/tablet, approval no.: H12020686, and price: 0.0869 CNY/tablet), and Etoposide (manufacturer: Qilu Pharmaceutical Co., LTD., specification: 5 ml:0.1 g/piece, approval no.: National Drug approval WORD H20143143, and price: 7.79 CNY/piece).e2.4. Outcomes' Index

#### 2.3.1. Treatment Efficacy Index

According to the uniform efficacy standard of the International Myeloma Working Group (IMWG), the efficacy of the patients after each cycle of treatment was evaluated. Efficacy was divided into strict complete response (sCR), complete response (CR), very good partial response (VGPR), partial response (PR), disease stabilization (SD), disease progression (PD), and relapse after complete response (relapse after CR). Define therapeutic effectiveness = sCR + CR + VGPR. Adverse reaction indicators: the occurrence of peripheral neuritis in treated patients was tracked and recorded in this experiment.

#### 2.3.2. Cost Index

Total expenses = hospitalization expenses + examination expenses + medicine expenses, hospitalization expenses = bed expenses + nursing expenses, examination fee = ultrasound fee + radiation fee + laboratory fee, medicine fee = Chinese medicine fee + western medicine fee, average daily cost = total expenses/days of hospitalization, and average treatment cost per cycle = total cost/number of treatment cycles. In this pharmacoeconomic evaluation, we only considered direct medical cost among direct costs. Due to the complexity of patient sources, direct nonmedical costs, including patient meals, patient transportation, patient wage loss, and family care, were not included in the cost calculation [4, 5]. The two groups were compared using *t*-test for statistical differences, and *P* value less than 0.05 was considered statistically significant.

## 3. Results

### 3.1. Baseline Characteristics of Included Patients

There was no statistical significance in gender, age, disease staging (ISS stage, traditional DS stage, and revised R-ISS stage) [6–8], and basic diseases (hypertension, diabetes, coronary heart disease, atrial fibrillation, cerebral hemorrhage, cerebral infarction, atherosclerosis, vein thrombosis of lower limb, hyperlipidemia, high uric acid hematic disease, hypothyroidism, thyroid nodules, chronic respiratory system disease, digestive system diseases, rheumatoid immune-related diseases, history of orthopedic surgery, allergies, etc.) (*P* > 0.05). See Table 1, for details.

### 3.2. Comparison of Treatment Efficacy and Safety

#### 3.2.1. Comparison of Treatment Efficacy and Safety in All Patients

Evaluated efficacy after each cycle of treatment: the effective cases were summarized and statistically analyzed. There was no statistical difference between the original drug research group and the generic drug group. The statistical results of each cycle are shown in Table 2 (*P* > 0.05).

There was no statistical difference between the evaluation groups for each treatment cycle, indicating equivalence. The incidence of peripheral neuritis during treatment is shown in Table 3 (*P* > 0.05). There was no statistical difference in the incidence of peripheral neuritis among the included patients.

One hundred and twenty seven patients were in the newly treated original research drug group and 102 patients were in the newly treated generic drug group. The occurrence and grading of peripheral neuritis in the two groups were compared, and the specific comparison results are shown in Table 4 (*P* > 0.05). There was no statistical difference in the incidence of peripheral neuritis among the newly treated patients.

#### 3.2.2. Comparison of Efficacy according to Different Starting States

Subgroup comparative analysis was conducted for patients with different initial states of disease, and they were divided into initial treatment MM group and recurrence/progression MM group. The effective cases were summarized and statistically analyzed, and there was no difference between initial treatment MM group and recurrence/progression MM group. Statistical results of each cycle are shown in Table 5 (*P* > 0.05). There was no statistical difference in the comparison between the subgroups of the included patients according to their different initial states, and the subgroup analysis was still equivalent [9].

#### 3.2.3. Comparison of Efficacy in the Treatment of VRD Regimen

Each MM patient included in the experiment with each course of treatment was considered as a unit, and the highest number of treatments was VRD (Bortezomib + Lenalidomide + Dexamethasone) regimen, with a total of 323 treatment units. The partial data were still divided into VRD original research drug group and VRD generic drug group, and their curative effect evaluation was statistically analyzed. Among them, 145 patients in the original research drug group were treated with 88 patients above VGPR, and the effective rate was 60.69%. There were 178 patients in the generic drug group, and 94 patients were treated with VGPR or above. The treatment effective rate was 52.81%. The treatment effective rate between the two groups was 0.155, *P* > 0.05. In the subgroup analysis with VRD as the treatment plan, there was no statistical difference between the original drug group and the generic drug group, and the subgroup analysis was still equivalent. The statistical results are shown in Table 6.

#### 3.2.4. Cost-Minimization Analysis of Treatment Costs

There was no statistical significance of efficacy and safety between original research drug and generic drug Bortezomib; therefore, cost-minimization analysis can be used for pharmacoeconomic analysis. Excluding the cases participating in clinical trials and data loss, 11 cases in the original research drug group and 8 cases in the generic drug group, the remaining 138 cases in the original drug group and 112 cases in the generic drug group were analyzed and compared during hospitalization. The average daily cost and average cycle cost of patients in the two groups were compared. The average daily cost of the original research drug group was 2954.38 CNY, and the average daily cost of the generic drug group was 2697.29 CNY, (*P* < 0.05). The average treatment cost per cycle was 32967.69 CNY, and the average treatment cost per cycle was 29129.57 CNY, (*P* < 0.05). The price of the average daily cost and the average treatment cost per cycle in the generic drug group were lower than the original drug group. Therefore, the generic drug group is more economical. The results were shown in Table 7.

## 4. Discussion

Our study results showed that there was no statistical significance of efficacy or safety between original research drug and generic drug Bortezomib. Compared with the original research drug, the generic drug has an obvious price advantage. Currently, the treatment of multiple myeloma is mainly induced by the proteasome inhibitor Bortezomib combined with glucocorticoid, plus the “three-drug combination” regimen with the immunomodulator thalidomide or lenalidomide, until autologous stem cell transplantation or disease progression [10, 11]. The treatment can obviously prolong the survival time and improve the quality of life. In application of Bortezomib for MM which is inevitable in the process of adverse reaction, hematology-related adverse reactions are mainly for neutropenia and nonhematology-related adverse reactions mainly include peripheral neuritis and cardiac toxicity [12, 13] and also include other herpes zoster, gastrointestinal reaction, paralytic ileus, venous thrombosis, and severe infections [14]. However, in all serious adverse reactions, peripheral neuritis has been confirmed to be the key factor for the dose limitation of Bortezomib application [15, 16]. It has a clear evaluation criterion, which has a significant effect on patients' life. Other serious adverse reactions require symptomatic treatment, which can be indirectly reflected in the treatment cost. In this study, the effectiveness of Bortezomib was compared between the original study and the generic Bortezomib, and there was no statistical difference between the groups. The collected data were used for subgroup analysis and were divided into initial treatment MM group and recurrence/progression MM group; there was no statistical difference of efficacy comparison between the groups. The effectiveness of all extracted drugs was compared between the original research drug and generic drug using VRD regimen, and there was no statistical difference between the groups. At the same time, the safety of the drugs was analyzed and compared. By comparing the occurrence of peripheral neuritis between the original research drug and generic drug in all the included patients, it was concluded that there was no difference in the occurrence of peripheral neuritis between the two groups. There was no difference in the occurrence of peripheral neuritis between the two groups. In summary, in this study, the efficacy and incidence of peripheral neuritis of the original and generic Bortezomib were analyzed and compared through multiangle and multi-subgroup analysis, which can prove that there is no difference in the efficacy and safety of the generic and the original research drugs in China, which can provide strong support for clinical drug selection.

In the data of this experiment, the average daily cost of the original research drug was 257.09 CNY/day higher than that of the generic drug, and the average treatment cost per cycle was 3838.12 CNY/cycle higher. The unit price difference of the two drugs was 1710.03 CNY/dose. Four doses of Bortezomib were applied in each cycle, and the difference was 6840.12 CNY/cycle, which was less than the difference of average treatment cost per cycle. There was a difference of 0.17 days/cycle between patients in hospital, indicating that the price difference was not completely derived from Bortezomib. The expenses included were hospitalization expenses, examination expenses, and drug expenses. It can be seen that, in the case of small hospitalization time difference, the drug expenses of Bortezomib original research group, the main chemotherapy drug, were 6,840.12 CNY/cycle higher than the generic drug group. The price difference of 6840.12 CNY/cycle -3838.12 CNY/cycle = 3002 CNY/cycle may be derived from the examination fee during hospitalization and the drug fee for symptomatic treatment when adverse reactions occur. Although part of the treatment cost of the original research drug group was lower than that of the generic drug group, the overall treatment cost of the generic drug group was significantly lower than that of the original research drug group.

There were also some limitations in our experiment, such as limited sample size and record content amd short tracking record time. In order to get more accurate conclusions, it is still necessary to accumulate more cases, conduct long-term follow-up, and establish an accurate database.

Compared with America and Japan, the consistency evaluation of generic drugs in China started late. However, China is a big country of generic drugs; about 95% or above chemicals are generic drugs. It can be seen that it is important for Chinese national health to obtain generic drugs with high purity of active ingredients, good stability, and good safety. In 2018, the National Medical Products Administration issued the Notice on Matters Related to The Consistency Evaluation of Generic Drug Quality and Efficacy and, in May 2020, issued a series of technical guidelines, including The Technical Requirements for consistency Evaluation of Generic Drug Quality and Efficacy of Chemical Injections, to further carry out the consistency evaluation of generic drugs in China. Nowadays, more and more generic drugs are coming to people's side, and the threshold of generic drug consistency evaluation should be strictly regulated so that people can use high-quality and inexpensive drugs [17].

The Harvard Business School Management Professor Michael Porter puts forward the concept of “value-based healthcare.” Different countries and teams have different interpretations of value-based healthcare. Under the social environment with serious aging trend of population, high incidence of chronic diseases, and rising medical costs, how to solve the “difficult and expensive medical treatment” has been a concern of the country, hospitals, and the masses. For patients with multiple myeloma, it is the embodiment of value medicine to improve the consistency evaluation standard of domestic generic drugs, ensure the effectiveness and safety of Bortezomib, reduce the price of generic drugs, improve the quality of life for patients with chronic cancer, and strive for longer survival time and material support.

## 5. Conclusion

We compared the original research drug and the generic drug Bortezomib in the treatment of MM. There was no difference between the two groups of effectiveness or safety, and the generic drug is more economical in treatment.

## Figures and Tables

**Table 1:** Comparison of baseline date in included patients.

	Original research drug group (*n* = 149)			Generic drug group (*n* = 120)			*P*
Median age	61			61			0.466
$\overset{¯}{X}$ ± S	60.55 ± 9.434			60.33 ± 8.665			

*Gender*							
Male	88 (0.59)			66 (0.55)			0.503
Female	61 (0.41)			54 (0.46)			

*Basic disease species*							
No basic disease	35 (0.23)			15 (0.13)			0.068
1 basic disease	41 (0.28)			28 (0.23)			
2 basic diseases	33 (0.22)			25 (0.21)			
3 basic diseases	20 (0.13)			29 (0.24)			
4 basic diseases	8 (0.05)			13 (0.11)			
5 basic diseases	5 (0.03)			5 (0.04)			
6 or more basic diseases	7 (0.05)			5 (0.04)			
Disease staging	I	II	III	I	II	III	
ISS	37 (0.25)	36 (0.24)	71 (0.48)	24 (0.20)	25 (0.21)	68 (0.57)	0.359
DS	5 (0.03)	16 (0.11)	125 (0.84)	5 (0.04)	14 (0.12)	98 (0.82)	0.902
R–ISS	14 (0.09)	58 (0.39)	29 (0.19)	13 (0.11)	51 (0.43)	28 (0.23)	0.435

**Table 2:** Comparison of treatment efficacy and safety in included patients.

Treatment cycle	Original research drug group			Generic drug group			*P*
	>=VGPR	Sample	Total efficacy rate (%)	>=VGPR	Sample	Total efficacy rate (%)	
1	20 (0.13)	149	13.42	22 (0.18)	120	18.33	0.270
2	44 (0.30)	149	29.53	31 (0.26)	120	25.83	0.501
3	80 (0.54)	147	54.42	65 (0.57)	114	57.02	0.676
4	92 (0.66)	139	66.19	75 (0.71)	105	71.43	0.383
5	91 (0.66)	137	66.42	69 (0.73)	95	72.63	0.315
6	90 (0.67)	134	67.16	71 (0.79)	90	78.89	0.056

**Table 3:** Comparison of peripheral neuritis among the included patients.

Peripheral neuritis	Original research drug group	Generic drug group	*P*
Cases	59	42	0.439
Incidence rate	39.60%	35.00%	

**Table 4:** Comparison of peripheral neuritis grades in newly treated patients.

Peripheral neuritis grade	Newly treated original research drug group (*n* = 127)	Newly treated generic drug group (*n* = 102)	*P*
1	9 (0.07)	7 (0.07)	0.595
2	20 (0.16)	10 (0.10)	
3	13 (0.10)	10 (0.10)	
4	0	0	

**Table 5:** Comparison of efficacy according to different starting states in included patients.

Subgroups	Treatment cycle	Original research drug group			Generic drug group			*P*
		>=VGPR	Sample	Total efficacy rate (%)	>=VGPR	Sample	Total efficacy rate (%)	
Initial treatment MM	1	17 (0.13)	127	13.39	21 (0.21)	102	20.59	0.145
	2	38 (0.30)	127	29.92	30 (0.29)	102	29.41	0.933
	3	72 (0.57)	126	57.14	62 (0.63)	98	63.27	0.354
	4	82 (0.68)	121	67.77	69 (0.76)	91	75.82	0.200
	5	80 (0.67)	119	67.23	63 (0.78)	81	77.78	0.105
	6	79 (0.71)	111	71.17	62 (0.82)	76	81.58	0.105

Recurrence/progression MM	1	3 (0.14)	22	13.64	1 (0.06)	18	5.56	0.397
	2	6 (0.27)	22	27.27	1 (0.06)	18	5.56	0.072
	3	8 (0.38)	21	38.10	3 (0.19)	16	18.75	0.202
	4	10 (0.56)	18	55.56	6 (0.43)	14	42.86	0.476
	5	11 (0.61)	18	61.11	6 (0.43)	14	42.86	0.305
	6	11 (0.85)	13	84.62	9 (0.64)	14	64.29	0.228

**Table 6:** Comparison of efficacy in the treatment of VRD regimen.

Subgroups	>=VGPR	Sample	Total efficacy rate (%)	*P*
VRD original research drug group	88	145	60.69	0.155
VRD generic drug group	94	178	52.81	

**Table 7:** Comparison of treatment costs for each cycle in included patients.

	Groups	Cases	Average	Standard deviations	Standard error mean	*P*
Average daily cost	Original research drug group	138	2954.38 CNY/day	955.22	81.31	0.044
	Generic drug group	112	2697.29 CNY/day	1053.41	99.54	

Average treatment cost per cycle	Original research drug group	138	32967.69 CNY/cycle	16374.99	1393.93	0.044
	Generic drug group	112	29129.57 CNY/cycle	12957.72	1224.39	

Average cycle length of stay	Original research drug group	138	12.52 days	6.67	0.57	0.816
	Generic drug group	112	12.35 days	3.90	0.37	

## Data Availability

The data used to support the findings of the study can be obtained from the corresponding author upon request.
